# Effect of Early Rehabilitation and Nursing Intervention on the Rehabilitation Prognosis of Elderly Stroke Hemiplegia Patients in the Department of Neurology

This article has been retracted.

**DOI:** 10.1155/2022/4958044

**Published:** 2022-03-15

**Authors:** Min Ning, Fang Chen, Hui Wu, Haihua Zheng, Chunmei Zheng, Shufen Li

**Affiliations:** ^1^Hainan Cadre Nursing Home (Hainan Geriatric Hospital) Rehabilitation Department, China; ^2^Hainan Cadre Nursing Home (Hainan Geriatric Hospital) Nursing Department, Haikou, Hainan 571100, China

## Abstract

**Objective:**

To explore the influence of rehabilitation outcomes in older patients with stroke hemiplegia from the neurology department by early rehabilitation nursing.

**Methods:**

70 cases of old patients with stroke hemiplegia from 2020/01 to 2021/01 were randomly divided into observation group (35 cases) and control group (35 cases). The control group was nursed by usual care. The observation group was nursed by early rehabilitation nursing. Nursing efficacy was observed.

**Results:**

The scores of active demand, resistance, and rehabilitation nursing cooperation degree after the nursing for the observation group were higher than the control group (*P* < 005). The score of NIHSS after the nursing for the observation group was lower than that for the control group (*P* < 005). The scores of BI, BBS, and Fugl-Meyer after the nursing for the observation group were higher than those for the control group (*P* < 005). The total rate of nursing satisfaction for the observation group was higher than the control group (*P* < 005).

**Conclusion:**

Early rehabilitation nursing can improve rehabilitation initiatives, rehabilitation outcomes, and nursing satisfaction in older patients with stroke hemiplegia from the neurology department.

## 1. Introduction

Stroke is a common disease in neurology, often in the elderly group, and has the characteristics of high disability rate and mortality rate. Paraplegia is a common sequel to stroke. Patients take decreased muscle strength, adverse activity, or inactivity of one limb as the main manifestations, which seriously affect their quality of life [1]. Clinical studies have shown that the optimal rehabilitation period for elderly patients with stroke hemiplegia is within 3 months after the onset. To maximize the help of patients to reduce sequelae and improve exercise function, experts point out that early rehabilitation intervention is necessary [2]. However, long-term repetitive treatment and boring rehabilitation exercises are easy to lead to resistance, and the cooperation of patients is also significantly reduced, leading to difficulty to guarantee rehabilitation prognosis [3]. Given the above situation, our hospital has summarized a set of early rehabilitation and nursing intervention strategies combined with many years of nursing experience, and the implementation effect is satisfactory. It is now summarized as follows.

## 2. Material and Methods

### 2.1. General Information

The 70 elderly patients with stroke hemiplegia were admitted to the Department of Neurology in January 2020 to approximately January 2021 were included as the subjects of this study. They were divided into two groups of 35 cases each, according to the random number table control method. The observation group included 19 men, 16 women, 60~78, average (66.42 ± 4.33), hemiplegia position: 20 left, 15 right and control group: 17 women, 60~78, average (67.16 ± 4.54), hemiplegia position: 21 left and 14 right. There was no statistically significant difference in the above baseline data between the two groups (*P* > 005). New-onset constipation that occurred within the first 4 weeks was determined in this study. Patients with new-onset constipation at 4 weeks were compared with others without constipation for any association with stroke outcomes at 12 weeks. The study protocol was approved by the local ethical committee for clinical research, and all procedures involving the participant were conducted according to institutional guidelines in compliance with the regulations. Both oral and written informed consents were obtained from all participants.

### 2.2. Inclusion and Exclusion Criteria

Inclusion criteria are as follows: meet the diagnostic criteria for stroke hemiplegia, no physical dysfunction before onset and be able to take care of themselves, no cognitive or communication impairment, and sign informed consent. Exclusion criteria are as follows: delirious, transient cerebral ischemia, and other limb dysfunction.

### 2.3. Methods

The control group received routine care, including condition monitoring, distribution of health knowledge manuals, medication guidance, and rehabilitation training.

The observation group received an early rehabilitation care intervention: (1) Cognitive care: publicize the relevant knowledge of disease and rehabilitation to patients through one-to-one explanation, organize the watch of health knowledge videos, and patiently answer patients' questions, so as to reduce their inner anxiety and depression, and reduce the sense of resistance to rehabilitation care, and encourage and care more for them, introduce successful experiences, improve patients' confidence in treatment, and enhance their enthusiasm for rehabilitation.(2) Language functional rehabilitation care: formulate the individualized language function exercise content according to the patient's condition, and gradually help the patients to train the oral expression ability and hearing, to exercise the brain to promote the recovery of neural function.(3) Motor function rehabilitation care: basic rehabilitation training should be carried out within 2 weeks after the onset, aiming to prevent related complications, posture management, affected limb massage, and passive activities and start active bed rehabilitation exercises during the soft paralysis period (including turning over, sitting position, hand function exercises, and lower limb flexion exercises), to increase the acting ability. The spastic period should be gradually needed to form a normal movement mode, which can be achieved by sitting conversion, standing balance training, walking training, etc. The recovery period is mainly to correct the incorrect exercise methods, improve the hand function, gait practice, and so on.(3) Daily life ability exercise: guide patients to conduct daily life behaviors such as dressing, eating, and grooming, at first can be assisted by nurses or parents and then gradually completed by patients independently, to improve their self-care ability.

### 2.4. Observing Indicators

Both groups were compared with rehabilitation enthusiasm before and after the intervention, including the National Institutes of Health Stroke Scale (NIHSS) score, Barthel index (BI) score, motor function changes, and care satisfaction.

Rehabilitation enthusiasm using our hospital homemade questionnaire evaluation content includes positive demand, resistance, rehabilitation care degree, and three aspects all use the percentage score; the resistance is negative score; the higher the score said the less resistance; the rest is of the positive score; the higher the score said more positive demand, the better the rehabilitation care cooperation.

The NIHSS score [4] includes language, facial paralysis, consciousness level, and gaze function, with the total score of 45 points; the higher the score indicates the worse the degree of nerve defect.

The BI score [5] includes the toilet, transfer, eating, modification, and other 10 items, with a total score of 100 points; the higher the score means the stronger the daily life activities.

The motor function was scored using the Berg Balance Scale (BBS) [6], and limb motor function (Fugl-Meyer) score [7] was conduct for the evaluation. The BBS score includes 14 related items including starting from the seat, standing without support, sitting without back seat, and sitting from standing, with a total score of 56 points; the higher the score indicates better balance function. The Fugl-Meyer score included a total of 17 items related to the upper and lower limbs, with a total score of 100. The higher the score, the better the patient's limb motor function. The flow chart of this study was as Figure 1.

Nursing satisfaction was assessed by using our homemade questionnaire, including communication ability, nursing service attitude, nursing operation skills, and nursing service quality. The total score was 100. The score above 90 was very satisfied, 60~89, and less than 60, and total satisfaction was calculated.

### 2.5. Statistical Analysis

The data were all statistically and processed using SPSS 22.0. *P* < 005 indicates a significant difference.

## 3. Results

### 3.1. Comparison of Rehabilitation Enthusiasm between the Two Groups

The positive demand scores, resistance, and rehabilitation care coordination scores were higher than that before the intervention, and there were significant differences between the groups (*P* < 0.05). The positive demand scores, resistance, and rehabilitation care coordination scores were higher than the control group, with significant differences between data comparison (*P* < 0.05), see Table 1.

### 3.2. Comparison of NIHSS and BI Scores between the Two Groups

Both groups with NIHSS scores were lower than those before intervention and higher BI scores than those before intervention. There were significant differences between groups (*P* < 0.05), observed groups after the intervention had higher BI scores than controls, as shown in Table 2.

### 3.3. Comparison of Motor Function between the Two Groups

BBS and Fugl-Meyer scores were higher after intervention than those before the same group, with a significant difference between data (*P* < 0.05). BBS and Fugl-Meyer scores after in the observed groups were higher than those in the control. Significant differences between data comparisons (*P* < 0.05) are shown in Table 3.

### 3.4. Comparison of Care Satisfaction between the Two Groups

The total satisfaction with care in the observed group was higher than in the control group, with significant interdata contrast differences (*P* < 0.05), as shown in Table 4.

## 4. Discussion

Stroke is a common acute cerebrovascular disease, with the characteristics of sudden onset, rapid progress, and many sequelae; hemiplegia is one of the common sequelae and is also the main reason for the limited physical control ability and reduced living ability after the onset of the disease. The survey shows that even if stroke patients have received timely and effective treatment, there is still a high incidence of hemiplegia [8]. How to reduce the incidence of hemiplegia through effective rehabilitation care interventions and improved patient rehabilitation prognosis is discussed.

Domestic research reports pointed out that to promote the gradual recovery of limb function in stroke hemiplegia patients, it needs to rely on the functional reorganization of the brain, which is closely related to the good plasticity in the central nervous system, and this plasticity is mainly manifested in the multi-level regulatory ability of the brain [9, 10]. Some experts also believe that the cerebral cortex of stroke patients has strong functional plasticity and functional reorganization. Through scientific and effective motor intervention, it can help to regulate and promote cortical plasticity, improve cerebral blood circulation, and promote the functional recovery of stroke patients with hemiplegia [11]. Some research reports also confirmed that patients with stroke hemiplegia will activate a large number of neurons when performing certain kinetic energy, and the gradual motor recovery is conducive to promoting the recovery of nerve and central function and reproducing the original lost function of the body [12, 13].

In this case, our hospital combines years of nursing experience to summarize a set of early rehabilitation nursing intervention strategies to correct incorrect cognition of rehabilitation nursing through cognitive nursing, reduce resistance, and improve rehabilitation enthusiasm; rehabilitation care to help patients improve language and physical function and daily life exercise to promote early rehabilitation was needed. Levy's [14] research reports show that implementing early rehabilitation care is conducive to improving patient compliance and reducing resistance. The results of this study show that the positive demand score, resistance score, and rehabilitation nursing cooperation score after intervention are higher than that of the control group, which also confirms that the implementation of effective nursing intervention is conducive to improving the rehabilitation enthusiasm of patients, which is extremely beneficial for the implementation of various rehabilitation nursing measures and ensure the nursing effect. In addition, the NIHSS scores were lower than the controls, and the BI scores, BBS scores, and Fugl-Meyer scores were higher than the controls, also indicating that the implementation of early rehabilitation care can significantly improve the rehabilitation prognosis of patients, which is related to many measures to improve patient neurological and motor function in early rehabilitation care, and on the other hand, it is also related to the improvement of the patient's rehabilitation enthusiasm [15]. The study report also confirmed that the implementation of early rehabilitation care can effectively improve limb function and quality of life in stroke hemiplegia patients, consistent with the results of this study. The overall satisfaction of nursing in the observation group was higher than in the control group, indicating that patients have a high recognition of early rehabilitation and nursing intervention, which is of positive significance for improving the overall quality of nursing services. However, there are also limits of this study. First, the number of patients is only 70, which is not enough. In further studies, there should be large number of patients, even in different clinical centers. Moreover, the assessment criteria are not abundant, which still needs more improvement. We believe the conclusion would be more substantial if the relevant indicators are followed up.

To sum up, early rehabilitation and nursing intervention can improve the rehabilitation enthusiasm of patients and improve the rehabilitation prognosis and nursing satisfaction, which deserves clinical recommendation.

## Figures and Tables

**Figure 1:** The flow chart of this study.

**Table 1:** Comparison of rehabilitation motivation between the two groups.

Grouping	Positive demand score		Resistance once score		Rehabilitation care coordination score	
	Before the intervention	After the intervention	Before the intervention	After the intervention	Before the intervention	After the intervention
Observe group (*n* = 35)	60.44 ± 7.07	82.93 ± 7.13	61.08 ± 6.33	84.42 ± 6.72	65.75 ± 7.11	88.17 ± 6.64
Control group (*n* = 35)	60.25 ± 7.15	71.36 ± 6.39	62.16 ± 6.95	70.25 ± 7.55	66.03 ± 7.59	72.06 ± 7.12
*t*	0.159	9.600	1.009	12.475	0.233	14.354
*P*	>0.05	<0.05	>0.05	<0.05	>0.05	<0.05

**Table 2:** Comparison of NIHSS scores and BI scores between the two groups.

Grouping	NIHSS score		BI score	
	Before the intervention	After the intervention	Before the intervention	After the intervention
Observe group (*n* = 35)	22.15 ± 3.43	9.12 ± 1.64	34.15 ± 5.07	83.26 ± 6.48
Control group (*n* = 35)	22.07 ± 3.28	14.65 ± 2.71	34.36 ± 5.13	63.35 ± 6.07
*t*	0.138	19.949	0.245	18.177
*P*	>0.05	<0.01	>0.05	<0.01

**Table 3:** Comparison of the motor functions of the two groups (scores, ±*s*)$\bar{x}$.

Grouping	BBS score		Full-Meyer score	
	Before the intervention	After the intervention	Before the intervention	After the intervention
Observe group (*n* = 35)	13.02 ± 3.22	37.21 ± 4.14	60.85 ± 5.77	88.26 ± 6.38
Control group (*n* = 35)	13.17 ± 3.15	30.53 ± 3.94	60.93 ± 5.81	73.47 ± 6.02
*t*	0.276	9.546	0.082	13.715
*P*	>0.05	<0.05	>0.05	<0.05

**Table 4:** Comparison of care satisfaction between the two groups.

Grouping	Very satisfied	Satisfaction	Not satisfied	Total satisfaction
Observe group (*n* = 35)	26 (74.29%)	8 (22.86%)	1 (2.86%)	34 (97.14%)
Control group (*n* = 35)	18 (51.43%)	11 (31.43%)	6 (17.14%)	29 (82.86%)
*χ* ^2^				3.968
*P*				<0.05

## Data Availability

The data used to support this study are available from the corresponding author upon request.
